The article "Comparative Study of Physical Education Teaching in Middle Schools at Home and Abroad Using Clustering Algorithm" was published in 2022. Journal: Comput Intell Neurosci.

# Comparative Study of Physical Education Teaching in Middle Schools at Home and Abroad Using Clustering Algorithm

**DOI:** 10.1155/2022/7277742

**Published:** 2022-06-18

**Authors:** Dejun Tan

**Affiliations:** Huizhou University, Huizhou 516001, China

## Abstract

Physical education in middle school is very important for teenagers, so it is also crucial to understand the differences between PET (Physical Education Teaching) systems in middle schools at home and abroad. The frontier and hotspot of PET research in middle schools at home and abroad are examined in this paper using citation analysis, information visualization, and cluster analysis, as well as CiteSpace software. The findings show that PET method research in China is qualitative, whereas PET method research in middle schools around the world is quantitative evaluation and empirical research. Domestic research hotspots focus on classroom instructional design, whereas foreign countries focus on load identification theory's application in instructional design. Frontier research in the United States is dispersed and covers a wide range of topics, whereas research in other countries focuses on cognitive load theory. The classification time of this improved algorithm is reduced by 190.97 seconds when compared to the traditional KNN algorithm, and the total time is increased by more than 50%. According to the findings, nonsports or nonsports influencing factors should be given more consideration in the study of adolescent physical fitness decline in China.

## 1. Introduction

Physical education is one way for schools to implement comprehensive education, and physical education in all levels and types of schools plays an important role in sports development. The purpose of the physical education curriculum is to assist students in mastering the fundamental theoretical knowledge of physical education as well as the fundamental skills of scientific exercise, as well as to establish a correct view of physical education, in order to achieve the goal of improving physical fitness and health. It can help us understand and discuss the interaction of various factors and their various forms in the overall process of Physical Education Teaching, which is conducive to dynamically grasping the essence and law of the process [1]. In general, there are many PET (Physical Education Teaching) systems in middle schools that can help to develop the teaching system in middle schools. Physical education is an important part of our country's middle school education, with a focus on the combination of physical education and fitness, as well as the function of leisure and entertainment [2]. With China's middle school physical education reform progressing, developing a scientific and effective middle school physical education model is becoming more important in addressing the practical issues that the current social environment imposes on the development of school physical education in the country. It is critical to study the PET model abroad because it is at the forefront of the development of high-level theory of school physical education.

The article "Comparative Study of Physical Education Teaching in Middle Schools at Home and Abroad Using Clustering Algorithm" was published in 2022. Journal: Comput Intell Neurosci.

PET mode is a teaching program that encapsulates a set of teaching principles. It consists of a relatively stable teaching process structure and teaching method system, which is primarily reflected in the design and implementation of units and teaching courses [3]. Teaching, according to Xiong et al. [4], is a step toward transforming learning experiences into units, courses, and procedures. Alternatively, it is the process by which teachers teach students to absorb knowledge and skills [4]. Alves et al. [5] believe that education is a form of social power and that knowledge allows some people to control others [5]. Oliveira et al. [6] believe that the social environment plays an important role in the development of children and that social activities can explain cognitive changes in children [6]. Learning, according to Barker et al. [7], is a process of reorganizing the cognitive system as well as a series of processes of acquiring knowledge from the media, imitating knowledge, and incorporating it into the knowledge framework [7]. It is stated that classroom learning motivation is a natural characteristic of students, not a result of teacher manipulation. By drawing concept maps, Kim et al. [8] developed a teaching tool to help us check whether students truly integrate new knowledge into their cognitive structure [8]. This methodology and conceptual relationship framework are extremely useful. PET theory and practice are linked by the fact that the PET model is not only theoretical but also operable. A comparison of Chinese and foreign PET models will aid us in absorbing the positive aspects of foreign PET models and serve as a useful reference for China's PET model reform.

Sports and PET are both effective ways to encourage teenagers' healthy development. Excellent PE teachers play a critical role in assisting students in developing their physical fitness, competitiveness, and self-confidence. Physical education majors bear the burden of training future physical education teachers, and the quality of that training is directly related to whether or not the training plan for undergraduate talents of physical education majors is scientific, reasonable, and in line with national conditions. The main goal of comparing PET schemes in middle schools in the United States and other countries is to see if foreign models and experiences can help improve the quality of domestic physical education professionals.

The article "Comparative Study of Physical Education Teaching in Middle Schools at Home and Abroad Using Clustering Algorithm" was published in 2022. Journal: Comput Intell Neurosci.

The main creative points of this paper are as follows: (1) By using the method of citation analysis, the knowledge maps of the development of PE teaching design in middle schools at home and abroad were constructed, respectively, and the development of PET design in middle schools at home and abroad was comprehensively compared and analyzed. By looking for the key nodes in the process of cluster analysis of cocited documents, this paper compares the key documents that have changed the research field in the history of PET design in middle schools at home and abroad in recent ten years. (2) Through the comparative analysis of physical training research at home and abroad, this paper finds out the shortcomings of physical training research in China and the gap between China and foreign countries, then provides new ideas and methods for the development of physical training in China, and at the same time provides some references for theoretical research of physical training in China.

## 2. Related Work

### 2.1. Study on PET

Brian et al. started with the concept of curriculum, pedagogy, and evaluation as interrelated school information system, put forward and discussed “quality sports” with curriculum, pedagogy, and evaluation as basic dimensions and the meaning of sports quality in each dimension, and thought that to realize quality education in PET, it is necessary to pursue and demonstrate quality education within and between curriculum, pedagogy, and evaluation [9]. Roure and Pasco [10] believe that physical ability is the athletic ability of the human body through the nerve-muscle system based on the energy metabolism of the three energy supply systems [10]. Ayers and Woods [11] regarded citation network as a directed acyclic network formed by a series of events and papers in time series, used a search algorithm to explore the events that can represent the mainstream direction and the connection paths that play a key role in the formation of citation network, and put forward the critical path algorithm in citation network [11]. Giordano and Christopher [12] pointed out that British universities implement the training goal of “thick foundation and wide caliber.” The training of sports talents in Japanese middle schools is adjusted and improved according to the social demand for sports talents [12].

Amatori et al. [13] pointed out that, with the change in social demand for sports talents, the training goal of physical education major in colleges and universities has changed from specialized training of physical education teachers to training comprehensive talents and applied talents with strong adaptability [13]. Li and Fan's [14] research focuses on the analysis of childhood feelings. It is necessary to carry out education, which is the way for every individual to feel the world [14]. Sui [15] thinks that the influence of social factors and cultural factors is very important in the personal learning process. It should be emphasized that people will internalize their social environment and their cultural expression in the process of learning [15]. Osborne et al. [16] have proved that physical education class is regarded as a secondary course in many middle schools, so it has not been highly valued, the teaching equipment of this course is backward, and the concern of leaders at all levels has not been fully implemented [16]. Garnham [17] believes that the rapid development of modern society has greatly improved people's living standards, people pay more and more attention to physical and mental health, and people's attention has gradually turned to physical exercise [17]. We should put the reform of physical education at the top of the government's education department and actively promote the reform of physical education.

The article "Comparative Study of Physical Education Teaching in Middle Schools at Home and Abroad Using Clustering Algorithm" was published in 2022. Journal: Comput Intell Neurosci.

### 2.2. Overview of Clustering Algorithm Research

Clustering algorithm [18, 19] has achieved remarkable results since it was applied to data mining analyzed some clustering methods from the perspective of data mining (such as strict distinction between similarity and distance measurement and relevant optimization criteria applied to clustering) put forward a method to determine the initial clustering center by using the neighbor information of data points, which also has a certain reference value. Chen and Qiu [20]used the multidimensional grid data structure of attribute space to divide the space into multiple cell grids [20]. According to different levels of resolution, it stores multiple levels of cell grids, which form a hierarchical structure, and each high-level cell grid is divided into multiple lower-level cell grids.

Qin et al. [21] proposed a method to automatically optimize parameters. Clustering algorithm based on a synchronous model can alleviate some difficult problems of clustering analysis and noise detection on traditional data and has the characteristics of dynamic, local, and multiscale analysis, which can solve the difficulties faced by clustering analysis of large-scale data to a certain extent [21]. Yang et al. [22] proposed a simple nearest neighbor clustering algorithm based on statistics, which can eliminate background noise and isolated points and detect clustering areas with different densities from some data sets [22]. Baracchini et al. [23] showed how to reduce the time cost of clustering algorithm by using the idea and method of nearest neighbor. This idea based on nearest neighbor can still be applied to the clustering method based on the synchronous model. Therefore, we think this problem has certain research significance [23].

The article "Comparative Study of Physical Education Teaching in Middle Schools at Home and Abroad Using Clustering Algorithm" was published in 2022. Journal: Comput Intell Neurosci.

## 3. Methodology

### 3.1. Design of Clustering

Data mining technology has been widely used in finance, commerce, medicine, and other fields. In recent years, educational informatization has been popularized continuously. It is an inevitable trend to develop data mining technology in the field of education, analyze these complicated educational data, study teachers' teaching methods, and improve students' learning effect. Applying data mining analysis technology to analyze and predict mixed teaching behavior in middle schools and providing powerful decision-making or guidance for teachers and learners is the focus of current research, and it is also a realistic problem to be solved urgently. Data mining is a process of extracting data information that meets different business objectives and feeding back the information to users based on massive data analysis. In order to obtain potentially effective information to meet the needs of users, it is necessary to fully tap the surface information, remove redundant data, and display key data to users intuitively. Prediction and description are two goals of data mining. Prediction refers to the use of some information fields and variables in the database to predict hidden useful information, and description refers to the description of data into understandable patterns.

Because clustering is done without knowing the data structure of data pattern, it is difficult to judge what is a good transformation of feature space and the selection of feature subset. In fact, for some data sets, one standard can produce good results, while other data sets show the opposite results. The problem of pooling high-dimensional data comes from different angles. Besides designing new dimensionality reduction algorithms, we should also study the integration method of dimensionality reduction of high-dimensional data.  Figure 1 shows the general steps of this method.

Clustering consists of two parts: set constructor ∏ and consensus function Γ. For a given data set, the set constructor generates a set of clustering schemes, and the consensus function analyzes and processes multiple clustering schemes of the set and finally outputs an optimized clustering scheme.

When there is a certain degree of linear correlation between variables in matrix *X*, the change of data *X* will be mainly reflected in the direction of the first few load vectors, and the projection of data matrix *X* on the last few load vectors will be very small, which is mainly caused by measurement noise. In this way, the matrix *X*_*s*_ can be written into the following formula after principal component decomposition:

(1) $$\begin{array}{c} X_{s}=t_{1}p_{1}^{T}+t_{2}p_{2}^{T}+\cdots +t_{k}p_{k}^{T}+E={\hat{X}}_{s}+E, \end{array}$$

where *E* is the residual matrix, which represents the change of *X* in the direction of *p*_*k*+1_ to *p*_*m*_ load vector, and it explains the measurement noise and model error factors. If only the reserved *k* principal component vectors (*k* < *m*) are used to reconstruct the original data, the estimated data matrix ${\hat{X}}_{s}$ and residual matrix *E* can be expressed as

(2) $$\begin{array}{c} {\hat{X}}_{s}=\sum_{i=1}^{k}t_{i}p_{i}^{T},\\ E=\sum_{i=k+1}^{m}t_{i}p_{i}^{T}. \end{array}$$

The consensus function analyzes and processes according to the pooled set to generate the final pooled result. Because there is no clear correspondence between groups in a cluster and those supervised set combination methods cannot be directly applied, it is difficult to combine cluster sets.

The article "Comparative Study of Physical Education Teaching in Middle Schools at Home and Abroad Using Clustering Algorithm" was published in 2022. Journal: Comput Intell Neurosci.

There are two advantages of using the consensus function to partition graphs in this section:

1. Graph division has a good learning area, and the algorithm of clustering to spectrum has been successfully applied in a large number of applications.
2. When calculating the weight of edges in a graph, the clustering set gives a simple and effective measurement method to define similarity, which is a prerequisite for the success of graph division.

For simplicity, we only use the grouping set part of this method. In the process of building a cluster set, every time the base clustering algorithm is executed, a similarity matrix will be generated. Finally, all similarity matrices will be combined into a main similarity matrix to generate a similarity map. The graph is divided into several subgraphs, and each subgraph is connected and can be labeled as a group. The similarity matrix is constructed as follows according to the probability density function:

(3) $$\begin{array}{c} P\left(s_{j}|x_{i}\right)=\frac{p\left(x_{i}|s_{j}\right)\times P\left(s_{j}\right)}{\sum_{k=1}^{m}p\left(x_{i}|s_{k}\right)\times P\left(s_{k}\right)}, \end{array}$$

where *m* is the number of clusters, Σ_*j*_ is the covariance matrix of relative cluster *j*, and *u*_*j*_ is the mean value of data objects in cluster *j*. The probability includes two parts: input data and clustering results. Therefore, the density vector is a good method for similarity measurement.

The article "Comparative Study of Physical Education Teaching in Middle Schools at Home and Abroad Using Clustering Algorithm" was published in 2022. Journal: Comput Intell Neurosci.

### 3.2. Feature Selection and Dimension Reduction

The general method of feature dimension reduction is to evaluate each original feature with an evaluation function, calculate its weight, and select features with high weight to form feature subsets. The basic process is as follows (Figure 2).

1. Initially, the feature set includes all original features.
2. Calculate the evaluation function value of each feature in the feature set.
3. Sort features according to the value of the feature evaluation function.
4. Select the first *k* features as feature subsets.
5. According to the selected feature subset, the dimension of the text vector is compressed to simplify the representation of the text vector.

Generally speaking, the feature item set should have three characteristics: a complete feature item can truly represent the target content. According to the difference in feature vectors, objects can be distinguished from other documents. The dimension of the refined feature vector should be as small as possible.

The idea of possibility matching is to attach a membership function of the fuzzy set to each element in the sample based on the possibility theory so as to limit the evaluation values compatible with the elements, which represent the range values of attributes represented by atoms. The elements in the sample are described by a probability distribution, which indicates the inaccuracy and uncertainty of the data. The similarity of two samples is calculated by calculating the matching degree between sample objects.

Let the sample space be *U*, *p* ∈ *U*, *q* ∈ *U*, *μ*_*p*_(*u*) as the membership function of *p* and *π*(*p*) as the probability distribution of *p*, both of which are functions from *U* to [0,1]. In order to calculate the similarity between sample *p* and sample *q*, two measurement functions are introduced: possible similarity and necessary similarity.

The possible similarity of *p* to *q* is as follows:

(4) $$\begin{array}{c} f\left(p\right)=\pi \left(p,q\right)\\ =\underset{u\in p}{\text{Sup}}\min\left(\mu_{p}\left(u\right),\pi_{q}\left(u\right)\right). \end{array}$$

*f*(*p*) gives the possible similarity between sample *p* and sample *qq*, that is, the degree of matching between the set tone of values compatible with sample *p* and the set of sample *q* values.

The necessary similarity between *p* and *q* is as follows:

(5) $$\begin{array}{c} g\left(p\right)=N\left(p,q\right)=\underset{u\in p}{\text{Inf}}\max\left(\mu_{p}\left(u\right),1-\pi_{q}\left(u\right)\right). \end{array}$$

*g*(*p*) gives the degree of certainty of *p* − *q* compatible values, that is, the degree to which the set of possible values of *q* is contained by the set of *p* compatible values.

The article "Comparative Study of Physical Education Teaching in Middle Schools at Home and Abroad Using Clustering Algorithm" was published in 2022. Journal: Comput Intell Neurosci.

Probabilistic clustering analysis is the application of probabilistic matching in clustering analysis. Traditional fuzzy clustering analysis can be roughly divided into two categories: one is based on fuzzy equivalence relationships, and the other is based on fuzzy similarity relationships. A clustering method based on fuzzy equivalence relations is known as probabilistic clustering. When the sample space is a finite set, a fuzzy equivalence matrix represents the fuzzy equivalence relation, while a Boolean equivalence matrix represents the ordinary equivalence relation. The fuzzy equivalence matrix is then converted to a Boolean equivalence matrix, resulting in a clustering analysis process.

### 3.3. Text Classification of PET Research in Middle Schools at Home and Abroad

Because cluster analysis can aid in the exploration of unknown data structures, the results of its analysis can provide the best sample set for classification and other tasks and reduce the workload of empirical analysis such as manual annotation, and it has become the starting point for a series of data analyses. It is widely used in descriptive and predictive models to help analyze the known data structure. Clustering analysis and classification fall under the category of machine learning when it comes to developing a learning model. As a result, studying arbitrary family shape processing and large-scale text classification through clustering is extremely important from the perspective of machine learning.

Calculate the Euclidean distance or cosine similarity between the sample to be classified and the known training sample, find the *K* nearest neighbor texts with the closest distance or the greatest similarity to the text to be classified, and then judge the *K* nearest neighbor texts of the text to be classified according to the category of the text to be classified [19]. Considering the distance and angle between two vectors, the representative function is defined. The defined representative function is applied to KNN weight calculation instead of the category attribute function.

Let the known category of training text *d*_*i*_ be *C*_*j*_, and define the importance of *d*_*i*_ to category *C*_*j*_ as the representative function *u*(*d*_*i*_, *C*_*j*_), as shown in (6).

(6) $$\begin{array}{c} u\left(d_{i},C_{j}\right)=\frac{1}{\text{Dist}\left(d_{i},{\bar{C}}_{j}\right)}\times \text{Sim}\left(d_{i},{\bar{C}}_{j}\right), \end{array}$$

where ${\bar{C}}_{j}$ represents the center vector of category *C*_*j*_, which is to add all the text vectors of category *C*_*j*_ and then average them. $\text{Dist}\left(d_{i},{\bar{C}}_{j}\right)$ represents the Euclidean distance from the training text *d*_*i*_ to the center of the category *C*_*j*_ to which it belongs, and $\text{Sim}\left(d_{i},{\bar{C}}_{j}\right)$ is the cosine similarity between the training text *d*_*i*_ and the center of the category *C*_*j*_ to which it belongs.

The article "Comparative Study of Physical Education Teaching in Middle Schools at Home and Abroad Using Clustering Algorithm" was published in 2022. Journal: Comput Intell Neurosci.

The value of *K* is determined by the spatial distribution of all points and can only be adjusted by the experimental results. Common methods for calculating distance include cos distance and Euclidean distance. In this paper, the cos distance formula is used to calculate the distance. Assuming there is a vector *A*, *B*, the cos distance between them is calculated by the following formula:

(7) $$\begin{array}{c} D_{\cos}=\frac{A\cdot B}{\left|A\right|\cdot \left|B\right|}. \end{array}$$

*A*, *B* and the denominator is the product of the length of the vector *A*, *B*.

In this paper, the naive Bayes classifier is used for comparative experiments. It is a classification method based on the Bayes rule, which is expressed as follows:

(8) $$\begin{array}{c} P\left(h|D\right)=\frac{P\left(D|h\right)P\left(h\right)}{P\left(D\right)}. \end{array}$$

*P*(*h*) is the prior probability of assuming *h*, *P*(*D*) represents the prior probability of training data *D*, *P*(*D*|*h*) represents the probability of observing data *D* when *h* holds, and *P*(*h*|*D*) is called the posterior probability of *h*.

The category attribute function *y*(*d*_*i*_, *C*_*j*_) in the KNN algorithm will be replaced by the following formula:

(9) $$\begin{array}{c} y\left(d_{i},C_{j}\right)=\left\{\begin{array}{cc} u\left(d_{i},C_{j}\right), & d_{i}\in C_{j},\\ 0, & d_{i}\notin C_{j}. \end{array}\right. \end{array}$$

In the KNN text classification algorithm, the improved K-medoids algorithm is applied to cut the training text. In the classification process of the KNN algorithm, the representative degree *u*(*d*_*i*_, *C*_*j*_) is used to replace the category attribute function *y*(*d*_*i*_, *C*_*j*_). The flow of this improved algorithm is shown in Figure 3.

## 4. Experiment and Results

### 4.1. Analysis and Comparison of PET Research Hotspots at Home and Abroad

In this paper, CiteSpace software is used to analyze the literature data with similar themes. Because the research methods used in this paper (word frequency analysis and cocitation analysis) have certain requirements for references and keywords in literature data, this index mainly checks literature data and CSSCI, and the database does not contain bibliographic data. During the operation, 15 items of bibliographic information and related information were counted, as shown in Figure 4. These 15 items reflect the most concerned hot topics in the field of PET research abroad.

The article "Comparative Study of Physical Education Teaching in Middle Schools at Home and Abroad Using Clustering Algorithm" was published in 2022. Journal: Comput Intell Neurosci.

Among these 15 papers, the papers involved the research of the combination of self-determination theory and PET. Therefore, the self-determination theory is also one of the hottest research points in the field of PET research abroad. Emphasis is placed on the influence of language and behavior of PE teachers on students and their professional development. Physical education courses are also studied according to the characteristics of girls. It can be seen that the research field of PET abroad is biased toward women. The keyword frequency statistics in a specific period is the concentrated expression of the research focus in a specific field in that period. Therefore, keyword frequency is an important index to reveal research hotspots in specific fields. In this work, the information of 10 articles cited twice is counted, as shown in Figure 5. These 10 documents will reflect the most concerned hot topics in the field of PET research in China.

It can be seen that the research hotspots represented by keywords in the keyword cooccurrence network mainly focus on school physical education, physical education, physical education curriculum, middle school physical education, physical education teachers, PET methods, physical education concepts, traditional physical education, national physical education, physical education, and health curriculum standards and educational theories. This conclusion is generally consistent with the key research points reflected in the previous highly cited literature.

China's PET practice research should appropriately increase the research on sports from the perspective of public health. At present, the research on PET practice in China is mostly biased toward students' physical condition, and the research on sports from the perspective of public health should be appropriately increased. China's physical education curriculum survey should pay more attention to the details of the physical education class program. At present, China's physical education curriculum research tends to pay more attention to the standards or reforms of physical education and health curriculum and should appropriately increase the research on the details of physical education curriculum (such as students' physical activity level).

### 4.2. Comparative Analysis of Research Hotspots of PET Design in Middle Schools at Home and Abroad

Comparing the hot keywords at home and abroad, we can see that there are some similarities between them. The same hot field reflects the intersection of teaching design research at home and abroad, and it is also the mainstream research field at home and abroad. Due to the different degrees of attention paid to some hot keywords, the research enthusiasm and depth will be different (Figure 6).

The article "Comparative Study of Physical Education Teaching in Middle Schools at Home and Abroad Using Clustering Algorithm" was published in 2022. Journal: Comput Intell Neurosci.

From the ontology of instructional design, foreign countries pay more attention to the research of teaching strategies, while domestic countries pay more attention to the research of teaching methods and models. The frequency of attention to constructivism theory research in China is relatively high and central, while that in foreign countries is relatively low, which shows that the attention to constructivism theory in China is higher than that in foreign countries in the past decade. In addition, foreign countries gradually pay attention to the influence of emotional factors on students' learning effect, and the study of learning motivation is highly valued. However, the frequency of student-centered middle school students' hot words in China is only 7. In recent years, the domestic educational circles have vigorously advocated the design concept of constructivism, but in practice, the dominant position of students is often neglected.

Foreign countries focus on the research of teaching strategies, while domestic countries focus on the research of teaching methods and models. There are many discussions on the ontology of instructional design in China. At present, in the information age, informational instructional design and networked instructional design have become hot spots, while foreign countries focus on performance technology research.

Using the mutation word detection technology and CiteSpace software algorithm, combined with the time distribution characteristics of word frequency, keywords with high-frequency change rate are detected from subject words, which are called mutation words. Determine the frontier research and development trend of specific disciplines or fields. After importing the data into CiteSpace, 41 domestic variant words and 3 foreign variant words can be detected, and their time zone views can be obtained by running them separately. The statistics of variant words in domestic instructional design are shown in Figure 7. Statistics of variant words in foreign instructional design are shown in Table 1.

It is clear that domestic research has progressed in the area of exploration, which is consistent with the findings of other national researchers. Every year, hot research topics in instructional design are identified, but the research is not innovative. Since then, the focus of instructional design theory research has shifted to cognitive science, particularly distraction research, and no new research topics have emerged. When compared to domestic research, foreign boundary research, cognitive load, and distraction effect have not piqued domestic researchers' interest. More practical research closely related to national instructional design appears to be more important to national researchers. Localization of instructional design theory research entails combining foreign culture with traditional Chinese culture and social needs, as well as reconstructing and internalizing theoretical achievements in instructional design from other countries that do not meet China's needs. In reality, what exists is a theoretical system with Chinese characteristics. Teaching design research is inherently boring, and any research results necessitate the investment of time and energy by researchers, which can be exchanged through hard work. It is commendable that researchers pay attention to the latest trends, new theories, new models, and new technologies. The original research can be abandoned, and researchers must pay attention to the application of new hotspots.

The article "Comparative Study of Physical Education Teaching in Middle Schools at Home and Abroad Using Clustering Algorithm" was published in 2022. Journal: Comput Intell Neurosci.

Physical training is an important part of physical training. In recent years, some domestic scholars have conducted many valuable theoretical and empirical studies on the research status, existing problems, and future development trends of physical training, most of which are based on local conditions. There are relatively few researches on visual angle, subjective thinking, and qualitative analysis, as well as macroscopic understanding and quantitative analysis of physical exercise theory and practice at home and abroad. According to the visualization results, the keyword distribution of physical exercise research at home and abroad is drawn, as shown in Figure 8.

From the time distribution point of view, China's physical training research started late, but with the rapid development of modern competitive sports and the vigorous promotion of national fitness, China's physical training has undergone tremendous changes compared with the past. Foreign countries have a wide range of research objects on physical training, while China's research objects on physical training are relatively limited, mostly concentrated on a few elite athletes of various competitive sports.

The research field of physical exercise in China is mainly concentrated in the field of competitive sports. Compared with foreign countries, there is less research on physical training in other aspects such as mass fitness and national physique; that is, the development of physical training in competitive sports and mass fitness is uneven. Foreign countries pay more attention to the synchronous development of theory and practice, while domestic theoretical research of physical training lags behind practice, with competitive sports as the main theoretical research and certain repetitiveness of research contents. Pay attention to the physical health, mental health, and cognitive status of teenagers and the elderly in order to improve their physical health and quality of life. However, many empirical studies in China have the largest number of athletes among them, and their main purpose is to improve the recovery quality and achieve better quality of life and good results.

The article "Comparative Study of Physical Education Teaching in Middle Schools at Home and Abroad Using Clustering Algorithm" was published in 2022. Journal: Comput Intell Neurosci.

### 4.3. Performance Analysis of Clustering Algorithm

The experimental Chinese corpus is used, and the training set and the test set do not overlap. The selected text categories include 30 categories, like art, education, history, law, transportation, politics, and so on. The training text set contains 9809 texts, and the test text set contains 9813 texts. The comparison results of algorithm time performance are shown in Table 2.

It can be seen from Table 2 that, compared with the traditional KNN algorithm, the sorting time is reduced by 190.97, and the total time is increased by more than 50%. To sum up, compared with the traditional KNN algorithm, the improved KNN algorithm in this paper has a significant improvement in time performance.

## 5. Conclusions

In this study, the frontier and key points in the field of PET research in middle schools at home and abroad are investigated, scientometrics and clustering algorithms are comprehensively applied, and quantitative analysis and qualitative analysis are combined. Self-determination theory has been discovered to be one of the hottest research hotspots in the field of PET research in other countries. Physical education curriculum research in China has a tendency to focus on the standard or reform of physical education and health curriculum. The frequency and centrality of constructivism theoretical research in China are higher, whereas the frequency and centrality of constructivism research abroad are lower. Both at home and abroad, emphasis is placed on the methods, steps, and scheme design of the teaching process, with foreign countries placing a greater emphasis on teaching strategy research. Physical training research in China is primarily focused on competitive sports, and the development of physical training in competitive sports, mass fitness, and other areas is uneven. Foreign countries place a greater emphasis on the simultaneous development of theory and practice, whereas domestic physical training theoretical research lags behind practice. When compared to the traditional KNN algorithm, this algorithm reduces classification time by 190.97 seconds while increasing total time by more than 50%. Improving one's ability to face the educational world necessitates a large number of teaching resources in order to improve classroom teaching quality.

The article "Comparative Study of Physical Education Teaching in Middle Schools at Home and Abroad Using Clustering Algorithm" was published in 2022. Journal: Comput Intell Neurosci.

## Figures and Tables

**Figure 1:** High-dimensional data clustering set process.

**Figure 2:** Text feature selection.

**Figure 3:** Improved algorithm flow.

**Figure 4:** Literature of PET research hotspots abroad cocited network literature information.

**Figure 5:** Keyword frequency in periodical cooccurrence network.

**Figure 6:** Hot keywords at home and abroad.

**Figure 7:** Statistics of abrupt words in domestic instructional design automation.

**Figure 8:** Distribution of keywords in physical training research at home and abroad.

**Table 1:** Statistics of abrupt words in foreign instructional design.

Year	Rate ofmutation	Frequency	Keyword
2011	2.36	13	Curriculum practice
2012	2.88	21	Information-basedinstructional design

**Table 2:** Time performance.

Time/min	Before improvement	Before improvement
Training time	0	72.43
Classification time	346.58	155.61
Total time	346.58	228.04

## Data Availability

The data used to support the findings of this study are available from the corresponding author upon request.
